# The Immunomodulatory and Regenerative Effect of Biodentine™ on Human THP-1 Cells and Dental Pulp Stem Cells: In Vitro Study

**DOI:** 10.1155/2022/2656784

**Published:** 2022-09-02

**Authors:** Duaa Abuarqoub, Nazneen Aslam, Rand Zaza, Hanan Jafar, Suzan Zalloum, Renata Atoom, Walhan Alshaer, Mairvat Al-Mrahleh, Abdalla Awidi

**Affiliations:** ^1^Department of Pharmacology and Biomedical Sciences, Faculty of Pharmacy and Medical Sciences, University of Petra, Amman, Jordan; ^2^Cell Therapy Center, The University of Jordan, Amman, Jordan; ^3^School of Medicine, The University of Jordan, Amman, Jordan

## Abstract

**Background:**

Pulp tissue affected by deep caries and trauma can be protected by vital pulp therapies in which pulp regeneration success depends on the degree of pulp inflammation and the presence of regenerative signals. Reparative dentinogenesis requires dental pulp stem cell (DPSC) activity which can be stimulated by many bioactive molecules to repair the dentine, mediating a balance between the inflammatory response and the reparative events. Therefore, this study was performed in order to investigate the immune-inflammatory effect of Biodentine capping material on DPSCs and macrophages.

**Method:**

THP-1, a human monocytic cell line, was differentiated to macrophages, and flow cytometry was used to analyze the expressions of specific macrophage markers. LPS-mediated infection was created for macrophages and DPSCs followed by treatment with Biodentine. CBA array was used to investigate the cytokine secretion followed by qPCR. Migration potential of treated DPSCs was also determined.

**Results:**

Our results showed that THP-1 cell line was successfully differentiated into macrophages as shown by surface marker expression. CBA array and qPCR results showed that Biodentine-treated DPSCs and macrophages upregulated anti-inflammatory cytokines and downregulated proinflammatory cytokines. Also, Biodentine enhances the migration potential of treated DPSCs.

**Conclusion:**

Biodentine capping material mediated the polarization of M1 to M2 macrophages suggestive of tissue repair properties of macrophages and enhanced the anti-inflammatory cytokines of DPSCs responsible for dentine-pulp regeneration.

## 1. Introduction

Pulp tissue is the most important tissue for the development of the tooth, providing strength and vitality. Unfortunately, the pulp might get inflamed or lose its functionality and structural integrity when exposed to an external stimulus such as traumas, deep caries, and attrition or restorative treatments. As a result of such exposures, dental pulp cells start to differentiate into odontoblasts which are responsible for the reparative dentine formation, through increasing the secretion of dentine matrix proteins and inducing dentine mineralization [1]. However, when teeth lose their pulps, they also lose the sensation of environmental changes. Moreover, pulpless teeth start to lose their potential to regenerate the dentine which makes the progression of caries easier and unremarkable [2]. The pulp capping and pulpotomy named as “vital pulp therapy” play a major role in preserving and protecting the vital pulp from any external stimulus; hence, the protected pulp would be able to perform its function properly by forming the reparative dentine bridges which is an indicator of the success of pulp therapy [3].

Capping materials are designed to stimulate the dentinogenesis process in vital pulp therapy. These materials are required to be biocompatible, retain high physiochemical standards, and stimulate the formation of dentine and the differentiation of dental pulp cells [4]. Calcium hydroxide (CH) was the first pulp capping biomaterial to be announced in the clinical field of dentistry [5]. It showed high capacity to stimulate dentine regeneration and has antimicrobial features. Nonetheless, the use of CH has become limited in the practice due to its high solubility in the oral fluids and its inefficient sealing properties. Moreover, CH fails to adhere to the native dentine, which leads to formation of tunnels in dentine bridges [5, 6].

Recently, a new biomaterial has been introduced to the capping materials called mineral trioxide aggregate (MTA). In comparison with CH, MTA showed more favorable characteristics such as self-setting ability that improves the production of less porous dentine bridges with high thickness in a very fast rate [7]. Yet, from the clinical point of view, MTA showed some drawbacks and limitations. MTA is composed of tricalcium aluminate which is responsible for the discoloration of tooth after surgery [8]. Moreover, it has a long setting time, which renders the practical use of MTA inefficient [9].

Biodentine (BD) is a new bioactive dentine substitute composed of calcium silicate and possesses similar mechanical properties as dentine. The high density, low porosity, quick setting time, good biocompatibility, beneficial impact on the critical pulp cells, and capacity to promote reparative and tertiary dentine production are all characteristics of the BD cement [10, 11]. Similar to MTA, Biodentine (BD) can be applied in both dental crown and root treatments [12, 13]. The main uses of Biodentine are direct pulp capping and pulpotomy [14], root-end filling [12], cervical and radicular restorations [13], dentine regeneration, and sealing the communications between pulp space and periodontal ligament [12]. However, BD is superior to calcium hydroxide in terms of its physical and mechanical properties, including low porosity, high compressive strength, low solubility, high density, and superior capacity to seal to dentine [11]. BD's bridge is produced in a very well-arranged pattern, which is localized and organized at the damage site. Additionally, the quality of the produced dentine was significantly better than that of calcium hydroxide, as the orthodentin organization of Biodentine's dentine bridges was seen with very clear visible dentine tubules. Additionally, cells effectively secreting the structure displayed osteopontin and DSP expression, two important regulators of reparative dentine development, in addition to the formation of new blood vessels inside the dentine bridges, resulting in the generation of vasodentine [6, 15].

For in vitro cultures, Biodentine (BD) showed low cytotoxic effects and increased proliferation potential in cultures of pulp cells, osteoblasts, and periodontal ligaments [16–19].

Similar to MTA, in vivo studies showed that Biodentine initiated sufficient biological response, comparable to MTA. On the other side, Biodentine induces a moderate immunological response but plays a key role in modulating this inflammatory response over time [11, 20].

Generally, the pulp tissue of a healthy tooth is directly involved in the immunoreactivity with other immune cells such as macrophages, which originated from monocytes that are highly distributed through the pulp tissue in quiescent state. The use of capping biomaterials to treat caries can elicit immunological reaction, starting the inflammatory response and harboring of macrophages into the inflammation site [20–22]. The direct contact of macrophages with the biomaterial that is used in the filling process stimulates these immune cells to produce more cytokines leading to strong inflammation [23, 24]. The secretion of cytokines represents processes in repair and destruction [25]. The first step of inflammation after the use of the filling material is the secretion of proinflammatory cytokines, interleukin-1 (IL-1), interleukin-6 (IL-6), interleukin-1beta (IL-1*β*), tumor necrosis factor (TNF), monocyte chemoattractant protein (MCP), and macrophage inflammatory protein1 (MIP1) [24].

Hence, the analysis of the toxicological and immunological effect of BD is highly important in order to understand the immune-inflammatory effects of BD. Very few studies have investigated the immunological effect of BD on immune cells. Thus, the significance of our study is aiming to explore the immunological effects of BD when cocultured directly with human THP-1 derived macrophage immune cells, where this cell line is considered an ideal cell model to study the inflammatory response of BD by measuring the expression and secretion levels of released cytokines. Additionally, this study is aimed at evaluating the impact of BD on the migration, inflammation, and regeneration of pulp tissue, when BD was cocultured directly with dental pulp progenitor stem cells (DPSCs). Our null hypothesis was established that there was no difference in the immunomodulatory effect and regeneration potential of cells after exposure to Biodentine (BD).

## 2. Materials and Methods

### 2.1. Study Design

Two different cell types were used: THP-1 human monocytic cell line and dental pulp progenitor stem cells (DPSCs) for inflammation and regeneration experiments, as shown in Figure 1.

### 2.2. Cell Culture of THP-1

THP-1 human monocytic cell line (ATCC, USA) was cultured as previously described [26], in RPMI 1640 media (Hyclone, USA) containing 20% fetal bovine serum (Gibco, USA) in addition to 4.5 g/l D-Glucose (Sigma, USA) in a 5% CO_2_ incubator at 37°C; media exchange was performed every 2-3 days.

#### 2.2.1. Differentiation of THP-1 into Macrophages

The differentiation of THP-1 into macrophages was done as previously described [26]. Briefly, 2 × 10^5^ cells/ml of monocytic THP-1 cells were cultured in 24-well tissue culture plates (SPL, Korea) for 24 h. Following that, the differentiation was done by treating cells with 100 nM phorbol 12-myristate 12-acetate (PMA, Bio-Techne, USA) for the next 24 h. Cell adherence is an indicator of successful differentiation into macrophages; therefore, nonadherent cells were aspirated from the culture.

#### 2.2.2. Characterization by Flow Cytometry: Monocytes vs. Macrophages

In order to determine the variation in the immunophenotyping characteristics, the expression of several cell surface markers was measured before and after the differentiation of THP-1 into macrophages. Therefore, cells were collected and stained with the following markers: CD68-FITC (eBioscience, USA), CD14-PE-cy7 (BD Biosciences, USA), CD206-PE (BD Biosciences, USA), CD11b-PE (Bioscience, USA), HLA-DR-PerCPCy5.5 (BD Biosciences, USA), SSEA1-FITC (BD Biosciences, USA), CD117-PE (BD Biosciences, USA), CD49f-PE (eBioscience, USA), CD29-APC (BD, USA), and CD45-FITC (BD Biosciences, USA). FACSDiva 8 software and FACSCanto II (BD Biosciences, USA) were used to acquire the samples. Data were analyzed by using FlowLogic software (version 7.3, Australia).

#### 2.2.3. Activation of Macrophages by LPS and Biodentine

The differentiated macrophages were activated by treating cells with 1 *μ*g/ml lipopolysaccharide (LPS, Santa Cruz) for 24 h. Following that, medium was aspirated and fresh media containing 2 mg/ml of Biodentine were added for the next 24 h. Untreated cells were used as control. After that, media and cells were collected from both treated and control cells.

#### 2.2.4. Expression Profile of Macrophages by Flow Cytometry after Biodentine Activation

To explore the effect of Biodentine on the immunophenotype of LPS-treated macrophages, surface marker expression profile was evaluated by flow cytometry.

First, cells were harvested, collected, and stained with the following fluorinated antibodies: CD68-FITC (eBioscience, USA), CD14-PE-cy7 (BD Biosciences, USA), CD206-PE (BD Biosciences, USA), CD49F-PE (eBioscience, USA), CD29-APC (BD, USA), CD11b-PE (eBioscience, USA), HLA-DR-PerCPCy5.5 (BD Biosciences, USA), CD117-PE (BD Biosciences, USA), CD45-FITC (BD Biosciences, USA), and SSEA-FITC (BD Biosciences, USA), for 30 min at room temperature. Samples were acquired and analyzed with FACSDiva software version 8 on a FACSCanto II (BD Biosciences, USA) and FlowLogic software 7.3.

### 2.3. Isolation of Dental Pulp Stem Cells (DPSCs)

#### 2.3.1. Sample Collection

Human impacted third molars were collected from healthy donors aged 24-, 25-, and 29-year-old (*N* = 3). All donors were healthy without any medical complications. Additionally, the collected teeth were healthy (not infected) and free of any dental caries, and the redness of the pulp is an indicator of its viability.

#### 2.3.2. Cell Culture of DPSCs

Dental pulp stem cells (DPSCs) were isolated from human third molars, as previously described [27]. The obtained DPSC cells were incubated in a 5% CO_2_ incubator at 37°C, until reaching 70-80% confluence.

#### 2.3.3. Treatment of Dental Pulp Stem Cells (DPSCs) by LPS and Biodentine (BD)

DPSCs were activated by using lipopolysaccharide (1 *μ*g/ml LPS, Santa Cruz) for 24 h. Then, culture medium was replaced with fresh media containing 2 mg/ml of BD for further 24 h. Untreated cells were used as control cells. After the incubation period, media and cells were collected from both groups and stored at −80°C.

### 2.4. Quantification of Inflammatory Cytokine Cytometric Bead Array (CBA)

To evaluate the impact of Biodentine (BD) on the secretion of cytokines from macrophages and DPSCs, a panel of cytokines containing IL-6, IL-8, IL-10, TNF-*α*, IL-1*β*, and IL-12p70 was utilized and the corresponding proteins were measured via human inflammatory cytokine CBA (BD Biosciences, USA) by flow cytometry. Samples were analyzed as previously described [26].

### 2.5. Gene Expression (RT-qPCR)

To measure the impact of Biodentine (BD) on the expression of cytokines of treated macrophage cells and DPSCs on gene level, qPCR was performed.

First, BD-treated cells either THP-1 macrophages or DPSCs and their control cells were harvested and collected by using 0.25% trypsin EDTA (Gibco, USA). Then, RNA was extracted from treated cells and their control by using Trizol-hybrid method (Qiagen, USA). Q-PCR analyses were performed, as previously described [26]. Q-PCR was performed by using CFX96 (Bio-Rad, Hercules, CA, USA), with the following conditions: denaturing 95°C for 10 s, annealing 60°C for 15 s, and extension 72°C for 10 s, and repeated in a 35-PCR cycle. The fold change of the target gene was normalized compared to the differentiated macrophages (THP-1 cells stimulated with PMA only). Additionally, for DPSC-treated cell fold change of the target gene was normalized to DPSCs, which is not activated by LPS. The specific primer set used for analysis is listed in Table 1. Gene fold regulation was calculated by using the following equations:

(1) $$\begin{array}{c} \text{Activated sample}:∆\text{Ct}=\text{Ct GOI}-\text{Ct HKG},\\ \text{Reference sample}:∆\text{Ct}=\text{Ct GOI}-\text{Ct HKG},\\ ∆∆\text{Ct}=∆{\text{Ct}}_{\text{Treated sample}}-∆{\text{Ct}}_{\text{Reference sample}}.\\ \text{Gene fold regulation}=2^{-∆∆\text{Ct}}. \end{array}$$

GOI stands for gene of interest, and HKG stands for housekeeping gene.

### 2.6. Migration Experiment

#### 2.6.1. Wound Healing Assay (Scratch Assay)

The wound healing assay was performed as previously described [28]. Briefly, 2 × 10^5^ of DPSC cells (at P3) were seeded into 6-well culture plates (TPP, USA) until reaching 100% confluent monolayer. A starvation step was followed by adding serum-free medium to the 100% confluent cells for 24 h. Then, a scratch was made on the confluent layer of cells. Then, inflicted monolayers were washed with PBS to remove cell debris and then treated with 2 mg/ml of *α*-MEM containing Biodentine, in addition to the cell culture medium which is used as a control for 24 h. The inflicted cultured cells were observed using an inverted microscope (Axio Vert, Zeiss, Germany) to detect the differences in closure pattern at two different time points 0 and 24 h.

### 2.7. Statistical Analysis

The results were analyzed by GraphPad Prism and Microsoft Windows Excel to determine the statistical differences among all assays. For the expression profile of undifferentiated and differentiated cells (flow cytometry markers), *t*-test was performed between groups and statistical analysis was calculated for each marker. Additionally, the *t*-test was used for the secreted cytokines at protein level and gene fold regulation between the treated and control groups (significance assumed for ^∗∗∗∗^*p* < 0.00005, ^∗∗∗^*p* < 0.0005, ^∗∗^*p* < 0.005, and ^∗^*p* < 0.05).

## 3. Results

### 3.1. Differentiation of THP-1 Cells into Macrophages

To confirm the success of differentiation from monocytes into macrophages, surface marker expression profile was evaluated by flow cytometry. The expression profile of differentiated macrophages was distinguished from THP-1 monocytic cells. As shown in (Figure 2 and Table 2), the expression of the following markers CD11b, CD68, CD206, SSEA1, HLA-DR, CD14, CD117, CD29, CD45, and CD49f was significantly upregulated in the differentiated macrophages compared to THP1-monocytes (*p* < 0.05).

### 3.2. Activation of Differentiated Macrophages by LPS and Biodentine

Differentiated macrophages were activated by using LPS. Remarkably, CD68, CD11b, CD29, and CD14 were upregulated significantly after the activation of macrophages by LPS, while CD49f and HLA-DR were downregulated. Moreover, SSEA1 and CD206 showed no or negligible activation (Figure 3 and Table 2). However, after treating activated macrophages with Biodentine (BD), the expression profile of the obtained macrophages was evident. CD29, CD45, and SSEA1 were downregulated compared to the control untreated macrophages, whereas CD14, CD117, and CD49f were slightly upregulated. Furthermore, CD68, CD11b, CD206, and HLA-DR showed negligible activation (Figure 4 and Table 2).

### 3.3. Cytometric Bead Array (CBA) and Gene Expression

#### 3.3.1. For Treated Macrophages

For BD-treated activated macrophages, IL-12p70, IL-1*β*, and TNF-*α* were downregulated compared to the untreated control cells in a significant manner (*p* < ^∗∗∗^, *p* < ^∗∗∗^, and *p* < ^∗∗∗∗^), whereas IL-6 and IL-10 were upregulated significantly in BD-treated macrophage cells compared to the untreated control cells (*p* < ^∗∗^, *p* < ^∗∗^). However, BD-treated macrophages showed the same expression levels of secreted IL-8 cytokines without statistical significance when compared to the control cells (Figure 5).

At the gene level, our data showed a significant increase in the expression of the IL-10 and TGF-*β* compared to the control untreated group (*p* < ^∗∗∗^, *p* < ^∗^), while for IL-1*β*, IL-6, and IL-, a significant downregulation was detected in Biodentine-treated macrophages compared to the control untreated cells (*p* < ^∗∗∗^, *p* < ^∗∗^, and *p* < ^∗^). For TNF-*α* and IL-12P40, no significant difference was observed among the treated group and their control cells (Figure 6).

#### 3.3.2. Cytometric Bead Array (CBA) and Gene Expression for Treated DPSCs

Flow cytometric results of CBA for BD-treated activated DPSCs cells showed that IL-10 and IL-12p70 were significantly upregulated compared to the control untreated cells (*p* < ^∗∗^, *p* < ^∗∗∗^), while IL-1*β* and IL-6 were downregulated significantly when compared to the control untreated cells (*p* < ^∗∗^, *p* < ^∗^), whereas for TNF-*α* and IL-8, a nonsignificant expression was found as compared to the control cells (Figure 7).

From gene expression analysis, we can conclude that Biodentine-treated DPSCs demonstrate a significant downregulation of IL-6, IL-8, and IL-1*β* (*p* < ^∗∗∗∗^, *p* < ^∗^, *p* < ^∗∗∗∗^) as compared to untreated cells, while IL-10, TGF-*β*, and TNF-*α* were significantly upregulated in comparison to control cells (*p* < ^∗∗^, *p* < ^∗∗^, *p* < ^∗∗∗^). On the other hand, IL-12P40 did not show any significant difference (Figure 8).

### 3.4. Migration: Wound Healing (Scratch Assay)

The migration potential of BD-treated DPSCs (2 mg/ml of Biodentine) was performed by evaluating the wound infliction closure under the microscope. Interestingly, Biodentine was able to stimulate the healing process of inflicted DPSCs by decreasing the width of the wound (Figure 9).

## 4. Discussion

In vital pulp therapy, both inflammation and dentine-pulp regeneration are important processes in order to conserve the functionality and to maintain the viability of pulp tissue when the capping material is used in clinical application [30]. After the first step of inflammation, progenitor cells such as dental pulp stem cells (DPSCs) are required to start the regeneration of dentine-pulp complex [31], as these DPSCs are known with their high potential to regenerate and repair the dentine matrix [32, 33]. Therefore, the success of pulp regeneration relies on the presence of progenitor's cells that are responsible for pulp regeneration and the control of inflammation [30].

This study has evaluated the immunomodulatory effect of Biodentine (BD) pulp capping material on THP-1 macrophages and its role in stimulating the dentine-pulp regeneration when exposed to DPSCs (Progenitor cells) of the pulp tissue.

For THP-1 cells, our data showed the successful differentiation of these monocytes into macrophages based on the cell surface markers' expression as analyzed by flow cytometry, and these results are in alignment with a previous study [34]. Macrophages are important innate immune cells that are associated with two distinct types: a proinflammatory subset M1with prototypic macrophage functions such as inflammatory cytokine production and bactericidal activity and an anti-inflammatory subset M2 linked with wound healing and tissue repair processes [35]. It has been investigated that classically activated macrophages (M1) produce IL-6, IL-1, and TNF-*α* while alternatively activated (M2) macrophages produce IL-10 and TGF-*β* and are thought to be associated with tissue repair [36]. Therefore, in order to activate these macrophage cells, macrophages were treated with lipopolysaccharide [29] to mimic a situation where macrophages are encountered with pathogen-associated molecular patterns (PAMPs) that are responsible for the initiation of immunological responses [37].

In our study, the secretion of both IL-6 and IL-10 at the protein level was significantly increased, while that of IL-1*β*, Il-12p70, and TNF-*α* was significantly downregulated in LPS-activated macrophages that are treated with Biodentine compared to the untreated macrophages. At the gene level, we found that Biodentine-treated macrophages exhibited a downregulation of proinflammatory cytokines such as IL-8, IL-6, and IL-1*β* and an upregulation of anti-inflammatory cytokines, IL-10 and TGF-*β*.

In order to determine the immunological responses in *in vitro* culture, cells were exposed to the treatment; then, secreted cytokines were measured in cell culture media. IL-6 is an early released cytokine secreted in a time-dependent manner, starting at the beginning of inflammation, and decreases with time. Thus, its secretion is accumulated in the culture media, resulting in upregulating different signaling pathways that would affect the detected level of IL-6 [35]. Previously published in vivo studies conclude similar results regarding the expression of IL-6 [20, 38]. Additionally, the upregulation in the expression of IL-12 at gene level could be explained by the posttranslational modification, as IL-12p40 is a subunit of IL-12p70; thus, the activation of the latter cytokine requires the binding of two subunits IL-12p40 and IL-12p35 [39].

Interestingly, we found the same effect of Biodentine on the DPSCs after stimulating the progenitor cells with LPS and subsequent exposure to Biodentine. Quantification of the released mediators showed that Biodentine-treated DPSCs have a significant upregulation of the anti-inflammatory cytokine IL-10 and a downregulation of expression of the following proinflammatory cytokines at both protein and gene levels, IL-6, IL-8, and IL-1*β*. The picture for IL-12 and TNF-*α* was different, as the results at protein level and gene level were in disagreement. This discrepancy can be attributed to the inverse correlation or posttranslational modifications [35, 40].

It has been investigated that the different isoforms of TGF-*β* play multiple roles in the formation and repair of the dentine-pulp complex since it acts as a potent regulator for initiation and resolution of inflammatory responses [31, 41–43]. It has also been suggested that macrophage polarization is also driven by TGF-*β* expression [44]. Similarly, IL-10, an anti-inflammatory cytokine, decreases the production of proinflammatory cytokines such as IL-6 and CXCL-8 which in turn suppresses the immune response and limits the tissue damage [42]. In addition, it has been found that IL-10 is upregulated in inflamed pulps and odontoblast-like cells thereby not only initiating the pulp's response to invading bacteria but also minimizing the intensity of infections [45].

Moreover, clinically, BD was able to regenerate Biodentine bridges without any pain or inflammation; thus, it is considered more suitable for clinical application when compared to calcium hydroxide and MTA in respect of safety and new dentine formation in the pulp chamber and the continuous root formation [6, 15, 46, 47]. Interestingly, our results were consistent with these published studies.

Our results are in favor of these findings. Furthermore, we found that DPSCs treated with Biodentine have high migration potential at the injury site which is an indicator for the potential of Biodentine to stimulate the regeneration of the dentine. Hence, our null hypothesis was rejected.

This current study was performed in vitro; therefore, our future prospects will be oriented toward understanding the possible consequences and the therapeutic outcomes through *in vivo* experiments.

## 5. Conclusions

Our study sheds light on the importance of choice of the pulp capping material. It shows that Biodentine can influence complement activation by modulating the polarization of macrophages, can initiate the anti-inflammatory response to maintain the tissue homeostasis, and can enhance the migration potential of the DPSCs as a successful determinant of dentine-pulp regeneration.

## Figures and Tables

**Figure 1:** Study design of the work plan.

**Figure 2:** Flow cytometric (a) histograms and (b) statistical analysis of the expression of surface markers of THP-1 monocytes and PMA-THP-1-treated cells (macrophages) (^∗^*p* < 0.05).

**Figure 3:** Flow cytometric histograms (a) and the analysis of the fluorescence intensity (b) of the expression of surface markers of differentiated macrophages compared to LPS-activated differentiated macrophages (^∗^*p* < 0.05).

**Figure 4:** Flow cytometric (a) histograms and (b) the analysis of the fluorescence intensity of macrophages' expression markers after treatment with Biodentine (BD) for 24 h, compared to the control untreated macrophages (^∗^*p* < 0.05).

**Figure 5:** Measurement of the expression level of cytokines secreted by macrophage cells, activated with lipopolysaccharides, then treated with Biodentine (BD), compared to the control untreated group by using CBA by flow cytometry (^∗∗∗∗^*p* < 0.00005, ^∗∗∗^*p* < 0.0005, ^∗∗^*p* < 0.005, and ^∗^*p* < 0.05).

**Figure 6:** Measurement of the expression level of cytokines secreted by macrophage cells, activated with lipopolysaccharides [29], then treated with Biodentine (BD), compared to the control untreated group at the gene level by using qPCR (^∗∗∗∗^*p* < 0.00005, ^∗∗∗^*p* < 0.0005, ^∗∗^*p* < 0.005, and ^∗^*p* < 0.05).

**Figure 7:** Measurement of the expression level of cytokines secreted by DPSCs, activated with LPS, and treated with Biodentine (BD), compared to the untreated control group, by using CBA by flow cytometry (^∗∗∗∗^*p* < 0.00005, ^∗∗∗^*p* < 0.0005, ^∗∗^*p* < 0.005, and ^∗^*p* < 0.05).

**Figure 8:** Measurement of the expression level of cytokines secreted by DPSCs, activated with LPS, and treated with Biodentine (BD) and compared to the untreated control group, at the gene level by using qPCR. (^∗∗∗∗^*p* < 0.00005, ^∗∗∗^*p* < 0.0005, ^∗∗^*p* < 0.005, and ^∗^*p* < 0.05).

**Figure 9:** Scratch assay was evaluated on DPSCs treated with Biodentine (BD) to determine the effect of Biodentine on the migration potential of treated DPSCs, compared to the control untreated cells. Wound closure was observed under the inverted microscope (scale bar = 100 *μ*m).

**Table 1:** Primer set of inflammatory cytokines.

Gene	F	R
IL-10	GCCAAGCCTTGTCTGAGATGATCC	CATTCTTCACCTGCTCCACGGCC
IL-1*β*	CAGAAGTACCTGAGCTCGCC	AGATTCGTAGCTGGATGCCG
TGF-*β*	GCGCGAGATCCTCTCCATTT	AGGTCCAGCATGAACATGGG
IL12-p40	CATCTGCCTCTTCTTGTGGGT	GACTGGGTCCGAGGGATCTT
TNF-*α*	CATCTGCCTCTTCTTGTGGGT	GACTGGGTCCGAGGGATCTT
IL-6	GGCACTGGCAGAAAACAACC	GCAAGTCTCCTCATTGAATCC
IL-8	CTGGCCGTGGCTCTCTTG	CCTTGGCAAAACTGCACCTT
PPIA “cyclophilin A”	TCCTGGCATCTTGTCCATG	CCATCCAACCACTCAGTCTTG

**Table 2:** Flow cytometric results of macrophages' expression percentages (%) for surface markers for all groups.

	THP-1 (%)	Macrophages (%)	BD (%)	Control (%)
SSEA1	24.76	44.28	47.48	63.16
CD206	2.83	3.52	8.32	6.71
HLA-DR	4.04	36.82	24.73	13.98
CD14	87.53	96.04	98.80	99.53
CD117	0.24	0.64	5.62	1.84
CD29	97.41	98.04	98.06	98.93
CD45	92.06	99.19	91.65	97.49
CD49f	90.49	99.91	97.80	99.37
CD68	9.93	37.67	94.66	94.96
CD11b	87.52	69.86	98.92	97.17

## Data Availability

No data were used to support this study.
